# miR-124a Involves in the Regulation of Wnt/*β*-Catenin and P53 Pathways to Inhibit Abdominal Aortic Aneurysm via Targeting BRD4

**DOI:** 10.1155/2022/9241959

**Published:** 2022-01-21

**Authors:** Yunhui Li, Meifeng Lv, Mingshu Lu, Hongliang Guan

**Affiliations:** ^1^Department of Vascular Surgery, Jinan People's Hospital Affiliated to Shandong First Medical University, China; ^2^Pharmacy Department of Jinan Second Maternal and Child Health Hospital, China; ^3^Department of Vascular Surgery, Shandong Shanxian Central Hospital, China

## Abstract

**Background:**

Abdominal aortic aneurysm (AAA) belongs to a progressive, gradual aortic rupture, which can lead to death without surgical intervention. The key factors regulating the occurrence and progress of AAA are not clear. Increasing studies have indicated that microRNA (miRNA) plays an important role in cancer development. miR-124a serves as a tumor suppressor in several neoplasms, and its upregulation can greatly inhibit the life activities such as malignant growth and migration of tumor cells.

**Aim:**

The objective of this study is to explore the association of miR-124a with AAA and to uncover the regulated mechanism of miR-124a on AAA progression.

**Methods:**

The specimens from the AAA patients were used for observing the miR-124a expression, and human aortic endothelial cells (hAoECs) were treated with AngII to establish the AAA cell models. The quantitative reverse transcriptase-polymerase chain reaction (qRT-PCR), CCK-8, transwell assay, flow cytometry assay, and western blot were conducted to unearth the regulation mechanism of miR-124a on AAA, and the dual-luciferase reporter assay was employed to investigate the downstream target of miR-124a.

**Results:**

miR-124a was significantly downregulated in the whole blood of the patients, and the decreased miR-124a was also observed in AAA cell models. Overexpressing miR-124a could effectively inhibit the proliferation and migration and promote the apoptosis of the AAA cells. The dual-luciferase reporter assay confirmed that BRD4 was a downstream target of miR-124a, and BRD4 upregulation could obviously reverse the effects of miR-124a on the phenotype of AAA cells. Moreover, it was found that miR-124a could regulate the activities of Wnt/*β*-catenin and P53 pathways via targeting the BRD4.

**Conclusion:**

Our data suggested that miR-124a could regulate the activities of Wnt/*β*-catenin and P53 to suppress the AAA progression via targeting the BRD4.

## 1. Introduction

Abdominal aortic aneurysm (AAA) is a dangerous vascular disease, and more 90% mortality in the patients with AAA is related with the rupture of the tumor [1, 2]. Some patients with AAA may express atypical symptoms such as abdominal and back pains which may not be categorized as clinical features of AAA; thus, the symptoms of most patients have become serious when they are diagnosed by screening studies [3, 4]. At present, specific medicines and surgery intervention are available for AAA treatment. However, even with current techniques, the prognosis and over survival rate of the patients remain unsatisfactory [5]. Moreover, although many studies have delved into the pathogenic mechanism of AAA, few targets can be used in the development of a drug [6]. Thus, continued focus on exploring the robust molecular methods are still urgent events for AAA treatment.

Recently, increasing evidences have suggested that microRNAs (miRNAs) take great part in the development of AAA [7, 8]. miRNAs consisting of 18-25 nucleotides play biological roles in the cells via involving in the translation suppression of special proteins [9, 10]. The dysfunction of miRNAs has been contributed as a key cause, leading to the progression of multiple diseases ranging from inflammations to cancers. The visible difference of miRNA profiles exists in the blood mononuclear cells of the AAA patients and healthy people, and some miRNAs have been proven to be important participants for the progression of AAA [11, 12]. Hence, the intervention in miRNA expression has been gradually thought as promising therapeutic strategies for AAA. miR-124a, an abundant miRNA in the central neuron system, has been linked to tumor progression. miR-124a serves as a tumor suppressor in several tumors, and miR-124a upregulation can effectively inhibit the life activities such as malignant growth and migration of tumor cells [12]. One research has shown that the levels of miR-124a in the pathological whole blood of the patients are aberrant, suggesting the potential connection between miR-124a and AAA [13]. Nevertheless, the functions of miR-124a on the progression of AAA remain unknown.

This study focuses on investigating the role of miR-124a in the AAA and revealing the regulation mechanism of miR-124a on AAA, aiming at providing some references for AAA treatment.

## 2. Material and Methods

### 2.1. Specimen Preparation

The study was proved by the ethics committee of Jinan People's Hospital Affiliated to Shandong First Medical University. The whole blood specimens of 15 patients with AAA and 15 health subjects were used in this study. The blood of the patients was centrifuged (1000 × *g*) for 10 min at 4°C for preparation of the serums, and then, the serums were stored at -70°C.

### 2.2. Cell Culture and AAA Model Establishment

Human aortic endothelial cells (hAoECs) were used in this study. The cells were cultured with DMEM including 10% FPS, 100 U/ml of penicillin, and 100 *μ*g/ml streptomycin. The cells were cultured in incubators with 37°C and 5% CO_2_. The cells were treated with 1 *μ*M/l AngII to establish the AAA model in vitro.

### 2.3. Cell Transfection

The miR-124a mimics and negative control of miRNA (miR-NC) purchased from Generay Biotech (Shanghai, China) were used in this study, and pcDNA-BRD4 and control pcDNA designed and purified by Generay Biotech (Shanghai, China) were used to regulate the level of BRD4 in the cells. The cells were cultured in 6-well plates to 70% confluence, and then, the transfectants were added into each well. In short, 4 *μ*g of DNA, 100 pmol RNA, or 10 *μ*l Lipofectamine 2000 were, respectively, diluted with 250 *μ*l serum-free, and then, the mixtures were incubated for 5 min. The diluted transfectants were completely mixed and incubated with diluted Lipofectamine 2000 in equal volume at 25°C for 20 min. After that, the cells in each well were added with 500 *μ*l of the final mixtures and cultured for 24 hours.

### 2.4. qRT-PCR

The levels of miR-124a and BRD4 in the whole blood and cells were measured by qRT-PCR. Total RNA was isolated from serum samples using a miRVana PARIS kit (Ambion, Austin, TX, USA) according to the manufacturer's instructions. The cells treated with TRIzol reagent for extraction of total RNAs, and adherent cells were treated with trypsase before RNA extraction. After that, the total RNA in the extracts were transcribed as cDNAs by a PrimeScript® RT reagent Kit (Thermo Fisher, Massachusetts, USA). The primers of miR-124a and BRD4 synthesized by a PrimeScript® RT reagent Kit (Thermo Fisher, Massachusetts, USA) were used in the experiment. The reaction systems (10 *μ*l) of qRT-PCR were prepared according to the operational instruction of a KAPA qRT-PCR kit (Sigma-Aldrich, Missouri, USA). U6 was used as the endogenous controls. The following conditions were used: denaturation at 95°C for 3 min, followed by amplification for 40 cycles at 95°C for 12 s and at 53°C for 40s, and 70°C for 30s. The relative levels of miRNA or mRNA were calculated with the 2^−(*ΔΔ*Ct)^ method [14]. The primer sequences of miR-124a, BRD4, and U6 are listed in Table 1.

### 2.5. Western Blot

Total proteins in the cells were extracted by RIPA buffer (Thermo Fisher, Massachusetts, USA). BCA assay kit was used to measure the concentration of the extracts, and the results were used to adjust the concentrations of all extracts. 30 *μ*l of the extracts were added into the separating gels, and the proteins were separated by polyacrylamide gels. After that, the proteins in the gels were transferred on the polyvinylidene fluoride (PVDF) membranes by the wet transfer method. Subsequently, the membranes were blocked with 5% milk for 1 hour, and the primary antibodies of the proteins such as BRD4, Wnt, *β*-catenin, P53, and *β*-actin were used to incubate the related membranes overnight at 4°C. The next day, the membranes were washed with TBST for three times and then were incubated with the second antibodies for 1 hour. After washing with TBST for three times, the levels of the proteins were quantified by a chemiluminescence detection system. The antibodies were used as follows: anti-BRD4 (1 : 1000, ab2610136, Thermo Fisher, Massachusetts, USA), anti-Wnt (1 : 1000, ab11154198, Thermo Fisher, Massachusetts, USA), anti-*β*-catenin (1 : 1000, ab2533039, Thermo Fisher, Massachusetts, USA), anti-P53 (1 : 1000, ab11004789, Thermo Fisher, Massachusetts, USA), and anti-*β*-actin (1 : 1000, ab2223496, Thermo Fisher, Massachusetts, USA).

### 2.6. Migration Assay

The migration of the cells was observed by transwell assay. In brief, the upper chamber of the transwell chamber was coated with Matrigel, and 5 × 10^4^ cells were seeded in the upper chamber of each transwell. After incubation for 24 h, the cells were fixed by 4% paraformaldehyde and stained with 0.4% trypan blue. After that, the cells migrated into the lower chambers were counted in three 3 randomly selected areas under a microscope (Olympus, Tokyo, Japan).

### 2.7. CCK-8 Assay

The cells were seeded into 96-well plates. After 48 hours of transfection, the cells in each well were added with CCK-8 solution (Amyjet, Wuhan, China), and the blank wells only added with CCK-8 solution as the controls. After incubating for 4 hours, the absorbance value was measured at 450 nm by a microplate reader (Molecular Devices, Shanghai, China).

### 2.8. Dual-Luciferase Reporter Gene Assay

The mutant and wild 3′-UTR sequences of BRD4 were inserted into the pmirGLO luciferase reporter vectors. The vectors containing the mutant sequence and wild sequence of BRD4 were named as BRD4-mutant type (BRD4-mut) and BRD4-wild type (BRD4-wt), respectively. BRD4-mut and BRD4-wt were, respectively, transfected into HEK-293T cells along with miR-769 mimics or miR-NC, and then, the cells were incubated for 48 hours. Finally, the luciferase activity of HEK-293T was observed by a dual-luciferase reporter assay system.

### 2.9. Flow Cytometry Assay

SGC7901 cells were treated with trypsinase (0.25%, EDTA-free). The harvested cells were washed by ice phosphate-buffered saline (PBS) for 3 times. After that, 2 × 10^3^ cells were suspended by 5 *μ*l of ice Annexin V-FITC binding buffer (10 *μ*g/ml), and then, the cells were incubated in the dark for 10 min. Finally, 10 *μ*l of propidium iodide (PI 20 *μ*g/ml) was added into the cells, and the apoptosis levels of the cells were instantly observed by flow cytometry equipment (BD Biosciences, State of New Jersey, USA).

### 2.10. Statistical Analysis

All experiments were performed at least 3 times, independently. The data were analyzed by SPSS 20.0, and the figures were charted by GraphPad Prism 8.0. Chi-squared test or ANOVA with Tukey's post hoc test was used to calculate the difference between the groups. *P* < 0.05 meant that statistical significance existed in the two groups.

## 3. Results

### 3.1. miR-124a Was Downregulated in the Tumor Whole Blood and AAA Cell Model

To explore the role of miR-124a in abdominal aortic aneurysm, the expression difference of miR-124a in tumor and paracancerous whole blood was analyzed by qRT-PCR. The results showed that miR-124a was extremely downregulated in the whole blood of the patients compared with health subjects (Figure 1(a), *P* < 0.01). Moreover, compared with normal cells, the miR-124a was significantly downregualted in the AAA cell model compared with normal hAoECs (Figure 1(b), *P* < 0.01). Those observations suggested that miR-124a was related with the progression of AAA.

### 3.2. miR-124a Restrained the Progression of Tumor Cells

Given the aberrant expression of miR-124a in tumor cells, it hypothesized that miR-124a involved the regulation on the phenotype of tumor cells. To verify this hypothesis, the miR-124a mimics were transfected into AAA cell models, and CCK-8 assay, transwell assay, and flow cytometry were used to observe the effects of miR-124a on model cells. It was observed that the cells expressed low viability after transfecting with miR-124a (Figure 2(a), *P* < 0.01). The transwell assay showed that miR-124 significantly inhibited the migration ability of model cells (Figure 2(b), *P* < 0.01). Moreover, the increased apoptosis level of model cells was also observed in the cell with high miR-124a level (Figure 2(c), *P* < 0.01).

### 3.3. BRD4 Was a Target of miR-124a, and BRD4 Was Upregulated in Tumor Whole Blood and AAA Cell Models

To further reveal the downstream factors of miR-124a, TargetScan was used to predict the targets of miR-124a. It was found that BRD4 was one of the targets of miR-124a. The dual-luciferase reporter assay was used to test the binding effect of miR-124a and BRD4. The results showed that miR-124a could effectively act with the wild type of BRD4 compared with the mutant type of BRD4 (Figure 3(a), *P* < 0.01). In addition, the increased mRNA level of BRD4 was also observed in the tumor whole blood and AAA cell models, and it was also found that miR-124a was extremely upregulated in AAA cell models compared with normal hAoECs (Figures 3(b) and 3(c), *P* < 0.01).

### 3.4. BRD4 Could Rescue the Inhibition of miR-124a on Tumor Cells

Although miR-124a could directly target the 3′UTR of BRD4, whether BRD4 plays a key role in the regulation of miR-124a on tumor development remains unclear. In the next study, the miR-124a mimics and BRD4-expressed vectors were cotransfected into tumor cells to observe their effects on the cellular phenotype of tumor cells. The CCK-8 showed that the inhibited viability of tumor cells induced by miR-124a upregulation was reversed by BRD4 (Figure 4(a), *P* < 0.01). The transwell assay reflected that BRD4 could significantly rescue the weakened migration ability of tumor cells with high miR-124a level (Figure 4(b), *P* < 0.01). Besides, the decreased apoptosis levels of tumor cells were also observed in the cells cotransfected with miR-124a mimics and BRD4 compared with the cells only transfected with miR-124a mimics (Figure 4(c), *P* < 0.01). Those observations suggested that the inhibitions of miR-124 on the tumor were related with BRD4.

### 3.5. The Regulation of miR-124a on Tumor Involved in Wnt/*β*-Catenin and P53 Pathways

To further investigate the regulation mechanism of miR-124a on the tumor development, western blot was used to observe the activity changes in the related signal pathways. The results showed that miR-124a significantly inhibited the expressions of Wnt and *β*-catenin (Figure 5, *P* < 0.01). Moreover, the increased P53 level was also observed in the cells after transfecting with miR-124a mimics (Figure 5, *P* < 0.01). Besides, it was also found that the effects of miR-124a on the levels of Wnt, *β*-catenin, and P53 could be reversed by BRD4 (Figure 5, *P* < 0.01). Those observations suggested that miR-124a could regulate the activities of Wnt/*β*-catenin and P53 pathways via targeting BRD4.

## 4. Discussion

Despite tremendous efforts using traditional approaches to reduce the mortality and morbidity of AAA disease, the identification of the underlying causes as well as appropriate medical intervention remain a major clinical challenge [15]. New approaches in understanding and fighting AAA are needed. Because of the complex pathological mechanisms of aneurysm progression, and rupture, the general ways of designing drugs to target specific enzymes, cell surface receptors, or single proteins are insufficient to counter the situations above [16]. The discovery of an entirely new method of gene regulation through miRNAs and their validation as markers and modulators of vascular remodeling in pathological conditions provide new therapeutic pathways for developing innovative therapies [12, 17]. This study revealed the connection of miR-124a and AAA, and the regulation mechanism of miR-124a on the progression of AAA was also investigated.

Recently, accumulating evidences have pointed out that the dysfunction of miRNAs takes a momentous effect on advancing the development of cancer cells [18]. In this study, it was also found that miR-124a was significantly downregulated in the tumor whole blood and AAA model cells compared with normal whole blood and cells. Low miR-124a level has been identified as an independent event which confers the poor prognosis and survival rate of the patients with acute lymphoblastic leukemia [19]. Moreover, the previous study has demonstrated that miR-124a is evidently downregulated in the whole blood of the patients with glioblastoma, and its ectopic expression could effectively impede the migration activity of cancer cells [20]. The fact is that downregulation of a single miRNA, miR-124a, in this study could inhibit the abnormal proliferation and migration of tumor cells and thereby block the development of the tumor, which reflected the effective functions of individual miRNAs involved in complex physiological and disease phenotypes of the tumor.

miRNAs always serve as the blockers for mediating the transcription inhibition of proteins to take part in the life activities of the cells via targeting the 3′-UTR of the related mRNAs [21]. Zhang et al. have affirmed that decreased miR-194 is related with the malignant proliferation of abdominal aortic aneurysm, and KDM3A, a target of miR-194, serves as a tumor promoter which promotes the progression of the tumor via mediating the activation of BNIP3 [22]. miR-24 was shown to be a key regulator of vascular inflammation and AAA pathology. This report revealed chitinase 3-like 1 (Chi3l1) to be a major target and effector under the control of miR-24, responsible for regulating cytokine synthesis in macrophages as well as their survival, promoting aortic smooth muscle cell migration and cytokine production, and stimulating adhesion molecule expression in vascular endothelial cells [23]. miR-124a has been proved as a tumor inhibitor in glioma cells, and miR-124a can restrain the proliferation and migration of tumor cells via targeting IQGAP1. Considerations have been given in the intervention of miR-124a in abdominal aortic aneurysm via the transcription inhibition of key proteins; BRD4 was determined as the downstream targets of miR-124a by TargetScan. Moreover, the increased BRD4 was also observed in the tumor whole blood and cell lines. BRD4 serves as a tumor promoter in multiple cancers and takes part in the cellular activities to boost the incontrollable growth of tumor cells [24]. Recent evidence has further added the complexity of BRD4's role in cancer, indicating that this protein has additional nontranscriptional functions that affect processes such as DNA damage repair, checkpoint activation, or telomere homeostasis. BETi-mediated inhibition of these BRD4 noncanonical activities can significantly affect the growth and survival of cancer cells. The recent study has emphasized the tumor promoter role of BRD4 in breast cancer, and BRD4 silence could effectively reduce the transcriptional activation of SNAIL and then impede the progression of the tumor [25]. Besides, it was also found that BRD4 could obviously rescue the inhibited effects of miR-124a on AAA cells. The results showed that BRD4 inhibition evidently restrains the malignant growth, migration, and inflammation of multiple tumor cells. Zhao et al. have confirmed that BRD4 downregulation could effectively inhibit the viability, invasive ability, and migration of pituitary adenoma cells [26]. Therefore, it is suggested that miR-124a could inhibit the phenotype of AAA cells via targeting BRD4.

The dysfunction of signal pathways such as Hippo, Wnt/*β*-catenin, and P53 has been widely accepted as major reasons of cancer development, and the consideration has been given in the connection of miR-124a and the related pathways [27]. The results in this study determined that miR-124a upregulation significantly suppressed the activation of Wnt/*β*-catenin and promoted the expression of P53, while those phenomena could be reversed by BRD4 upregulation. In glioma stem cells, it has been confirmed that BRD4 could enhance the activity of the Wnt/*β*-catenin pathway via promoting the expression of miR-142-5p, and BRD4 has also been identified as a suppressor of P53 to promote the progression of acute myeloid leukemia [28, 29]. Hence, it suggests that miR-124a could inhibit the development of AAA via regulating the activation changes of Wnt/*β*-catenin and P53 pathways mediated by BRD4.

In this study, the evidences of miR-124a regulating the progression of AAA were provided; the downstream target and regulation mechanism of miR-124a on AAA were also investigated and illustrated by cell models. However, a limitation of the present study is that although miR-124a was identified as a regulator in AAA progression, we did not conduct more experimental studies to explore unknown functions of this miRNA in vivo and its interplay with other miRNAs that were expressed in AAA tissues.

## Figures and Tables

**Figure 1:** miR-124a was significantly downregulated in the whole blood of the patients and AAA cells. (a) The relative expression level of miR-124a in whole blood was measured by qRT-PCR. (b) The relative expression level of miR-124a in AAA cells was measured by qRT-PCR. ^∗∗^*P* < 0.01. AAA: abdominal aortic aneurysm.

**Figure 2:** miR-124a upregulation inhibited the proliferation and migration and promote the apoptosis of AAA cells. (a) The effect of miR-124a on the proliferation of AAA cells was observed by CCK-8 assay. (b) The effect of miR-124a on the migration of AAA cells was observed by transwell assay. (c) The effect of miR-124a on the apoptosis of AAA cells was observed by flow cytometry. ^∗∗^*P* < 0.01. AAA: abdominal aortic aneurysm.

**Figure 3:** BRD4 was a downstream target of miR-124a, and BRD4 was significantly upregulated in the whole blood of the patients and AAA cells. (a) The binding effect of miR-124a and BRD4 was observed by dual-luciferase reporter assay. (b, c) The relative mRNA levels of BRD4 in whole blood of the patients and AAA cells were measured by qRT-PCR. ^∗∗^*P* < 0.01. AAA: abdominal aortic aneurysm.

**Figure 4:** BRD4 upregulation reversed the effects of miR-124a on the phenotype of AAA cells. (a) The proliferation of AAA cells was observed by CCK-8 assay. (b) The migration of AAA cells was observed by transwell assay. (c) The apoptosis of AAA cells was observed by flow cytometry. ^∗∗^*P* < 0.01. AAA: abdominal aortic aneurysm.

**Figure 5:** miR-124a regulated the activities of Wnt/*β*-catenin and P53 pathways via targeting BRD4. (a) The relative expression levels of miR-124a in AAA cells were measured by qRT-PCR. (b–f) The relative expression levels of BRD4, Wnt, *β*-catenin, and P53 were measured by western blot. ^∗∗^*P* < 0.01. AAA: abdominal aortic aneurysm.

**Table 1:** Primer sequence of miR-124, BRD4, and U6.

Name of primer	Sequences
miR-124a-F	5′-GAGGGGAGGGGTCTGGAG-3′
miR-124a-R	5′-GCCCAGAGAAAAATCTGCAC-3′
BRD4-F	5′-GAGCTACCCACAGAAGAAACC-3′
BRD4-R	5′-GAGTCGATGCTTGAGTTGTGTT-3′
U6-F	5′-CTCGCTTCGGCAGCACA-3′
U6-R	5′-AACGCTTCACGAATTTGCGT-3′

## Data Availability

The data used during the present study are available from the corresponding author upon reasonable request.

## References

[1] Doyle B., All The A. (2021). Response to "re biomechanical assessment predicts aneurysm related events in patients with abdominal aortic aneurysm". *European Journal of Vascular and Endovascular Surgery*.

[2] Yang H., Zhou T., Sorenson C. M., Sheibani N., Liu B. (2020). Myeloid-derived TSP1 (thrombospondin-1) contributes to abdominal aortic aneurysm through suppressing tissue inhibitor of metalloproteinases-1. *Arteriosclerosis, Thrombosis, and Vascular Biology*.

[3] Doyle B. J., Bappoo N., Syed M. B. J. (2020). Biomechanical assessment predicts aneurysm related events in patients with abdominal aortic aneurysm. *European Journal of Vascular and Endovascular Surgery*.

[4] Arnaoutakis D. J., Scali S. T., Neal D. (2020). Surgeon experience association with patient selection and outcomes after open abdominal aortic aneurysm repair. *Journal of Vascular Surgery*.

[5] Xie T., Yin L., Guo D. (2021). The potential role of plasma fibroblast growth factor 21 as a diagnostic biomarker for abdominal aortic aneurysm presence and development. *Life Sciences*.

[6] Spear R., Boytard L., Blervaque R. (2019). Let-7f: a new potential circulating biomarker identified by miRNA profiling of cells isolated from human abdominal aortic aneurysm. *International Journal of Molecular Sciences*.

[7] Dong M., Gong L. P., Chen J. N. (2020). EBV-miR-BART10-3p and EBV-miR-BART22 promote metastasis of EBV-associated gastric carcinoma by activating the canonical Wnt signaling pathway. *Cellular Oncology (Dordrecht)*.

[8] Shen G., Sun Q., Yao Y. (2020). Role of ADAM9 and miR-126 in the development of abdominal aortic aneurysm. *Atherosclerosis*.

[9] Chen W. H., Luo G. F., Sohn Y. S., Nechushtai R., Willner I. (2019). miRNA-specific unlocking of drug-loaded metal-organic framework nanoparticles: targeted cytotoxicity toward cancer cells. *Small*.

[10] Eckstein M., Sailer V., Nielsen B. S. (2019). Co-staining of microRNAs and their target proteins by miRNA in situ hybridization and immunohistofluorescence on prostate cancer tissue microarrays. *Laboratory Investigation*.

[11] Wang J., Sun H., Zhou Y. (2019). Circular RNA microarray expression profile in 3,4-benzopyrene/angiotensin II-induced abdominal aortic aneurysm in mice. *Journal of Cellular Biochemistry*.

[12] Lareyre F., Clement M., Moratal C. (2019). Differential micro-RNA expression in diabetic patients with abdominal aortic aneurysm. *Biochimie*.

[13] Chang Z., Zhao G., Zhao Y. (2020). BAF60a deficiency in vascular smooth muscle cells prevents abdominal aortic aneurysm by reducing inflammation and extracellular matrix degradation. *Arteriosclerosis, Thrombosis, and Vascular Biology*.

[14] Li J., Yan S. (2021). MiR-466 inhibits the progression of severe hepatocellular carcinoma via regulating FMNL2-mediated activation of NF-*κ*B and Wnt/*β*-catenin pathways. *Journal of Oncology*.

[15] Lai C. H., Chang C. W., Lee F. T. (2020). Targeting vascular smooth muscle cell dysfunction with xanthine derivative KMUP-3 inhibits abdominal aortic aneurysm in mice. *Atherosclerosis*.

[16] Yu M., Chen C., Cao Y., Qi R. (2017). Inhibitory effects of doxycycline on the onset and progression of abdominal aortic aneurysm and its related mechanisms. *European Journal of Pharmacology*.

[17] Plana E., Galvez L., Medina P. (2020). Identification of novel microRNA profiles dysregulated in plasma and tissue of abdominal aortic aneurysm patients. *International Journal of Molecular Sciences*.

[18] Gan S., Pan Y., Mao J. (2019). miR-30a-GNG2 and miR-15b-ACSS2 interaction pairs may be potentially crucial for development of abdominal aortic aneurysm by influencing inflammation. *DNA and Cell Biology*.

[19] Agirre X., Vilas-Zornoza A., Jimenez-Velasco A. (2009). Epigenetic silencing of the tumor suppressor microRNA Hsa-miR-124a regulates CDK6 expression and confers a poor prognosis in acute lymphoblastic leukemia. *Cancer Research*.

[20] Fowler A., Thomson D., Giles K. (2011). miR-124a is frequently down-regulated in glioblastoma and is involved in migration and invasion. *European Journal of Cancer*.

[21] Li G., Cheng Z. (2021). miR-339-5p inhibits autophagy to reduce the resistance of laryngeal carcinoma on cisplatin via targeting TAK1. *BioMed Research International*.

[22] Zhang H., Wang Y., Bian X., Yin H. (2021). MicroRNA-194 acts as a suppressor during abdominal aortic aneurysm via inhibition of KDM3A-mediated BNIP3. *Life Sciences*.

[23] Maegdefessel L., Spin J. M., Raaz U. (2014). miR-24 limits aortic vascular inflammation and murine abdominal aneurysm development. *Nature communications*.

[24] Liang D., Yu Y., Ma Z. (2020). Novel strategies targeting bromodomain-containing protein 4 (BRD4) for cancer drug discovery. *European Journal of Medicinal Chemistry*.

[25] Lu L., Chen Z., Lin X. (2020). Inhibition of BRD4 suppresses the malignancy of breast cancer cells via regulation of Snail. *Cell Death and Differentiation*.

[26] Zhao P., Cheng J., Li B. (2021). lncRNA PCAT6 regulates the progression of pituitary adenomas by regulating the miR-139-3p/BRD4 axis. *Cancer Cell International*.

[27] Borges K. S., Pignatti E., Leng S. (2020). Wnt/beta-catenin activation cooperates with loss of p53 to cause adrenocortical carcinoma in mice. *Oncogene*.

[28] Latif A. L., Newcombe A., Li S. (2021). BRD4-mediated repression of p53 is a target for combination therapy in AML. *Nature Communications*.

[29] Song H., Shi L., Xu Y. (2019). BRD4 promotes the stemness of gastric cancer cells via attenuating miR-216a-3p-mediated inhibition of Wnt/*β*-catenin signaling. *European Journal of Pharmacology*.

